# Exosome-mediated lncRNA AFAP1-AS1 promotes trastuzumab resistance through binding with AUF1 and activating ERBB2 translation

This article has been retracted.

**DOI:** 10.1186/s12943-020-1145-5

**Published:** 2020-02-05

**Authors:** Mingli Han, Yuanting Gu, Pengwei Lu, Jingyi Li, Hui Cao, Xiangke Li, Xueke Qian, Chao Yu, Yunqing Yang, Xue Yang, Na Han, Dongwei Dou, Jianguo Hu, Huaying Dong

**Affiliations:** 1 Department of Breast Surgery, The First Affiliated Hospital of Zhengzhou University, Zhengzhou, 450052 China; 2 Department of Vascular Surgery, The First Affiliated Hospital of Zhengzhou University, Zhengzhou, 450052 China; 3 Department of Oncology, The First Affiliated Hospital of Zhengzhou University, Zhengzhou, 450052 China; 4 Department of General Surgery, University-Town Hospital of Chongqing Medical University, Chongqing, 400016 China; 5 Department of Obstetrics and Gynecology, The Second Affiliated Hospital, Chongqing Medical University, Chongqing, 400010 China; 6 Department of General Surgery, Hainan General Hospital, Hainan Affiliated Hospital of Hainan Medical University, No.19 XiuHua Road, Xiuying District, Haikou, 570311 China

**Keywords:** Breast cancer, Trastuzumab resistance, Exosome, AFAP1-AS1, ERBB2

## Abstract

**Background:**

Although trastuzumab provides significant clinical benefit for HER2-positive breast cancers, responses are limited by the emergence of resistance. Recent evidence suggests that long noncoding RNAs (lncRNAs) play important roles in tumorigenesis and chemoresistance. However, the regulatory mechanism of lncRNAs in trastuzumab resistance is not well established to date. In this research, we identified the differentially expressed lncRNA and investigated its regulatory role in trastuzumab resistance of breast cancer.

**Methods:**

LncRNA microarray and qRT-PCR were performed to identify the dysregulated lncRNAs. Transmission electron microscopy, differential ultracentrifugation and qRT-PCR were used to verify the existence of exosomal AFAP1-AS1 (actin filament associated protein 1 antisense RNA 1). Bioinformatics prediction, RNA fluorescence in situ hybridization (RNA-FISH) and immunoprecipitation assays were performed to identify the direct interactions between AFAP1-AS1 and other associated targets, such as AU-binding factor 1 (AUF1) and ERBB2. Finally, a series gain- or loss-functional assays were done to prove the precise role of AFAP1-AS1 in trastuzumab resistance.

**Results:**

AFAP1-AS1 was screened out due to its higher expression in trastuzumab-resistant cells compared to sensitive cells. Increased expression of AFAP1-AS1was associate with poorer response and shorter survival time of breast cancer patients. AFAP1-AS1 was upregulated by H3K27ac modification at promoter region, and knockdown of AFAP1-AS1 reversed trastuzumab resistance. Moreover, extracellular AFAP1-AS1 secreted from trastuzumab resistant cells was packaged into exosomes and then disseminated trastuzumab resistance of receipt cells. Mechanically, AFAP1-AS1 was associated with AUF1 protein, which further promoted the translation of ERBB2 without influencing the mRNA level.

**Conclusion:**

Exosomal AFAP1-AS1 could induce trastuzumab resistance through associating with AUF1 and promoting ERBB2 translation. Therefore, AFAP1-AS1 level may be useful for prediction of trastuzumab resistance and breast cancer treatment.

## Introduction

Breast cancer has become a leading cause of cancer-related deaths in the world, and the most common cancer among women [1, 2]. About 20% of breast cancer patients are overexpressed with HER-2 and therefore associated with poor prognosis [3]. Currently, trastuzumab, a humanized monoclonal antibody targeting extracellular region of HER-2, has become the alternative choice in the treatment of HER-2-positive breast cancer [4]. However, only a fraction of metastatic patients responds to trastuzumab and approximately 60% develop resistance after initial response [5].

Long noncoding RNAs (lncRNAs) constitute a large class of mRNA-like transcripts, greater than 200 nucleotides with no protein coding capability [6, 7]. They are involved in a large variety of biological processes, with reports linking the dysregulation of lncRNAs with cancer cell invasion, proliferation and metastasis through mechanisms ranging from transcriptional levels to post-transcriptional levels [8, 9]. Recently, various of studies have reported that lncRNAs are key regulators in trastuzumab resistance of breast cancer. For example, Li et al. demonstrated that lncRNA GAS5 suppresses trastuzumab resistance in breast cancer [10]. Zhu et al. reported that lncRNA UCA1 induces trastuzumab resistance by sponging miR-18a [11]. Shi et al. revealed the critical role of lncRNA ATB in trastuzumab resistance in breast cancer [12]. These studies suggest that lncRNAs may be important regulators in the formation of trastuzumab resistance, however, the detailed function and the involved regulation pathway are not well known.

Exosomes, which are membrane-derived vesicles that originate from endosomal multivesicular bodies, have a size range of 20-150 nm when released into the interstitial fluid. These vesicles contain protein, lipids, coding or noncoding RNAs derived from their donor cell cytoplasm and can be taken up by other cells [13]. Exosomes provide a relatively stable environment for the therapeutic agent of choice, have the potential to be modified to improve cell specific homing, and have the ability to fuse with the plasma membrane of cells allowing therapy to directly enter the cell [14]. Previously, we identified a series of lncRNAs (e.g. SNHG14 and TINCR), which play important roles during trastuzumab resistance in breast cancer [15, 16]. However, whether lncRNAs cause trastuzumab resistance of breast cancer cells and spread to receipt sensitive cells by packaging into exosomes is not well known.

In this study, we performed microarray-based gene expression profiling of trastuzumab-resistant breast cancer by using the established trastuzumab-resistant cells. We identified actin filament associated protein 1antisense RNA 1 (AFAP1-AS1), a 6.8-kb lncRNA that is located in the chromosome 4p16.1, was dysregulated and closely associated with resistance to trastuzumab therapy. Moreover, we proved the essential role of AFAP1-AS1 in trastuzumab resistance by incorporating into exosomes. Mechanically, AFAP1-AS1 could bind with AU-binding factor 1 (AUF1) protein, which enhanced the translation of ERBB2 gene.

## Materials and methods

### Patient samples

Overall, 64 HER-2 positive patients who received trastuzumab treatment and 40 HER-2 negative patients were enrolled in this study. The clinical pathological information was shown in Additional file 1: Table S1. Cancerous tissues were collected from January 2013 to August 2014 and snap-frozen in liquid nitrogen instantly at − 80 °C. In addition, serum samples from above 64 HER-2 positive patients were also collected to investigate the predictive role of serum AFAP1-AS1. Patients who received radiotherapy and chemotherapy before surgical treatment were excluded. Meanwhile, the general clinical information and detailed pathological records were collected. Written-informed consent was obtained from all patients and the study protocol was approved by the Research Scientific Ethics Committee of The First Affiliated Hospital of Zhengzhou University and Hainan General Hospital. The overall survivals of these patients were followed up with a median period of 35 months. Overall survival (OS) was calculated from the date of surgery to the date of mortality or the last follow-up. Progressive-free survival (PFS) was calculated from the date of surgery to the date of first recurrence or the last follow-up.

### Cell culture and treatment

Human HER-2-positive breast cancer cell lines SKBR-3 and BT474, were purchased from American Type Culture Collection (Manassas, United States) and maintained in Dulbecco’s modified Eagle (DMEM, HyClone Lab., Inc., Logan, UT) medium supplemented with 10% fetal bovine serum (FBS) (Sigma-Aldrich, St. Louis, MO, USA), 100 U/ml penicillin and 100 μg/ml streptomycin (Life Technologies, Grand Island, NY, USA) in humidified air at 37 °C with 5% CO_2_. The cell lines were authenticated by short tandem repeat (STR) profiling. Trastuzumab (Herceptin) was purchased from Roche (Basel, Switzerland) and used by dissolving in phosphate-buffered saline (PBS). The SKBR-3 and BT474 cells resistant to trastuzumab treatment (named as SKBR-3-TR and BT474-TR, respectively) were built by establishing xenografts followed by four courses of trastuzumab treatment as previously described [16]. Cycloheximide (CHX, Sigma Aldrich, cat. no. 01810) was used at a final density of 20 μg/ml for 1 h.

### Vector construction and cell transduction

The silencing RNA against AUF1 (si-AUF1), AFAP1-AS1 (si-AFAP1-AS1#1, si-AFAP1-AS1#2) and HNRNPA2B1 (si-HNRNPA2B1) were synthesized and purchased from GenePharma (Shanghai, China). Negative control siRNA is purchased from Invitrogen (CAT#12935–110, Carlsbad, CA, USA). AFAP1-AS1, HNRNPA2B1cDNA or negative control cDNA was enlarged and cloned into the pcDNA3.1 expression vector, defined as p-AFAP1-AS1 and p-NC. shRNAs targeting AFAP1-AS1 (sh-AFAP1-AS1) or negative control (sh-NC) were synthesized and loaded into lentivirus for in vivo assays. Lipofectamine 3000 (Invitrogen, Carlsbad, CA, USA) were used for transfection with the final concentration of 100 nM according to the manufacturer’s instructions. The sequences of small interfering RNAs are presented in Additional file 2: Table S2.

### Quantitative real-time polymerase chain reaction (qRT-PCR) analysis

Total RNA was extracted with TRIzol reagent (Invitrogen, CA, USA) and treated with DNase I (Thermo Scientific, Waltham, MA, USA). Exosomes were isolated using ExoQuick Exosome Precipitation Solution (SBI, CA, USA) and exosomal RNAs were extracted using miRNeasy Mini Kit (Qiagen, Valencia, CA) followed by converting into cDNA using random primers and Revert AidM-MuLV reverse transcriptase (Thermo Scientific). The cDNA templates were amplified by real-time PCR using the SYBR Green PCR Kit (TaKaRa, Tokyo, Japan). qRT-PCR was conducted on an Applied Biosystems 7500 Sequence Detection System (Applied Biosystems, Thermo Fisher Scientific, Inc.), and the thermal cycling conditions were as follows: 95 °C for 30 s followed by 45 cycles of 95 °C for 5 s and 60 °C for 30 s. The final extension was 72 °C for 5 min. The specific primers were listed in Additional file 2: Table S2. Experiments were repeated three times and the relative expression of RNA was calculated using2^-ΔΔCt^ method [17].

### Expression profile analysis of lncRNAs

SKBR-3-TR and SKBR-3 cells were used for screening the differentially expressed lncRNAs. Five samples were enrolled for both groups. The extraction of total RNA, sequencing platform, data analyzation and the construction of cDNA library were done as previously described [16].

### Cell viability assay

The ability of cell proliferation was detected by CCK-8 (Dojindo, Kumamoto, Japan) according to the manufacturer’s instructions. A total of 5000 cells with corresponding treatment were seeded onto 96-well culture plates. At specific time point, CCK-8 reagent was used for incubation for 2 h at 37 °C. Then, the absorbance at 450 nm was determined by the Infinite M200 spectrophotometer (Tecan, Switzerland).

### EdU incorporation assay

The transfected breast cancer cell lines were put on sterile coverslips in 96-well plates and incubated for 2 days. EdU kit (RiboBio, Guangzhou, China) was used in line with user guidebook. The fixed cells were subjected to 0.5%TritonX-100 (Beyotime Inc., Shanghai, China) for 10 min and Apollo reaction for 30 min. Nuclei double-staining with EdU and 4′,6-diamidino-2-phenylindole (DAPI; Beyotime) were seen as positively proliferative cells.

### Cell migration assay

To determine cell migration, after transfection, 1 × 10^4^ cells were plated in medium without serum in the top chamber of a Transwell (Corning), while the medium containing 20% FBS was placed in the lower well. After 24-h incubation, cells were fixed by 4% formaldehyde for 15 min, the using crystal violet dye staining for 20 min and photographed under 100× magnification by a microscope. Experiments were carried out at least three times.

### Exosomes isolation

Exosomes in breast cancer cell culture supernatant were purified by differential ultracentrifugation. Briefly, cells were cultured in DMEM supplemented with 10% exosome-depleted FBS (SBI, CA, USA) for 48 h, then cell culture supernatant was collected and spun at 2× 10^3^g for 20 min, 4 °C to remove cells and 1× 10^4^g for 30 min, 4 °C to remove cellular debris. The resulting supernatant was filtered through 0.2 μm filters (Millipore), followed by ultra-centrifugation at 1× 10^5^ g for 1 h under 4 °C. The pellets were resuspended in PBS and ultra-centrifuged again at 1× 10^5^ g for 1 h under 4 °C. ExoQuick Exosome Precipitation Solution (SBI) was used to isolate exosomes from serum followed by exosomal RNA extraction using miRNeasy Mini Kit (Qiagen, Valencia, CA).

### Transmission electron microscopy (TEM)

Exosomes isolated as described above were used for ultramicroscopic analysis. Briefly, exosomes were resuspended and fixed in 30 μl 2% paraformaldehyde and adsorbed onto a glow-discharged copper grid. Afterwards, copper grid with exosomes adsorbed was suspended above the 3% glutaraldehyde droplet for fixation then suspended above the 4% uranyl acetate droplet to stain exosomes. Image capture was executed with TEM (FEI, United States).

### RNA immunoprecipitation (RIP) and chromatin immunoprecipitation (ChIP)

RIP was implemented using a Magna RIP™RNA-Binding Protein Immunoprecipitation Kit (Millipore, Cambridge, MA, USA) as directed by the manufacturer. Post the harvest of cells in IP lysis buffer and mechanical shear by a homogenizer, anti-bodies against AUF1 (cat. no. ab61193, Abcam, Cambridge, MA), HNRNPA2B1 (ab31645, Abcam) and IgG (EMD Millipore, cat. no. 12–371) were added and cultured with the cell extract overnight under 4 °C. Then streptavidin-coated magnetic beads were added for incubation for 2 h. The isolated and purified RNAs in which AFAP1-AS1 may be enriched was subjected to qRT-PCR measurement.

ChIP assay was carried out by the use of Simple ChIP® Enzymatic Chromatin IP Kit (Cell Signaling Technology, CA, USA). The cross-linked RKO and LOVO cell lines were cultured in 4%formaldehyde for 30 min at room temperature, followed by lysing in RIPA buffer (Thermo Scientific, Waltham, MA, USA). Lysates were treated with ultrasonic to acquire DNA fragments of 200- to 1000-bp in length. Immunoprecipitation was conducted with specific antibodies against H3K27ac antibody (Abcam, cat. no. ab4729) or the negative control IgG antibody (EMD Millipore, cat. no. 12–371) overnight at 4 °C. Following rinsing and elution, de-cross-linked chromatin was retrieved and quantitated by qRT-PCR with IgG antibody as negative control. Experimental procedures were performed at least 3 times.

### Nucleocytoplasmic separation

Nuclear and cytosolic fractions were separated using the PARIS kit (Am1921, Thermo Fisher Scientific, USA) as directed by the manufacturer. Then, the expression levels of GAPDH, U1 and AFAP1-AS1 in cytoplasm or nuclear of breast cancer cells were detected using qRT-PCR assay.

### RNA fluorescent in situ hybridization (RNA-FISH)

GFP-labeled AFAP1-AS1 probes were obtained from RiboBio. Hybridizations were carried out using FISH Kit (RiboBio Inc.) according to the manufacturer’s instructions. Briefly, 4% paraformaldehyde was used to fix the cardiomyocytes followed by the treatment of 0.5% Triton. Then, cells were cultured with specific probe overnight. All fluorescence images were captured using Nikon A1Si Laser Scanning Confocal Microscope (Nikon Instruments Inc., Japan). The sequence for AFAP1-AS1 probe is: 5′-ATTCCTTTATTTTATGGGATGTTCTGTAGGGAGTT-3′.

### Immunohistochemistry (IHC) analysis and scoring methods

Paraffin-embedded sections of tumor tissues from nude mice were placed in an incubator maintained at 60 °C for 2 h and then immersed. Used different concentrations of ethanol (including 100, 95, 85, 70%) and deionized water to hydrate these slices, then these slices were immersed in citrate buffer solution (0.01 mol / L, pH 6.0) and heated them and keep the temperature between 95 °C and 100 °C for 30 mins. After washing with PBS, incubated with 0.5% Triton X100 for 30 min. This fraction was then stained using the biotin-streptavidin HRP detection system (ZSGB, China). These slices were incubated with primary antibody targeting HER-2 (1:200, ab16901, Abcam) overnight at 4 °C, and the presence of brown chromogen in the membrane indicates positive immunoreactivity.

The immunostaining intensity of each sample was graded as negative = 0, weak = 1, moderate = 2, or strong = 3. The proportion of positively staining cells was assessed as the percentage. The score was then calculated as the intensity score multiplied by the percentage of cells stained (score = intensity × % of positive cells). Images were visualized using a Nikon ECLIPSE Ti (Fukasawa, Japan) microscope system and processed with Nikon software.

### In vivo nude mouse model

Tumor xenografts were established with male BALB/c nude mice (4–6 weeks old), which were purchased from Model Animal Research Center of Nanjing University (Nanjing, China). They were randomly divided into two groups of five each and housed three per cage in pathogen-free conditions at 28 °C, 50% humidity in a specific sterile environment suitable and regularly observed. A total of 3 × 10^6^ SKBR-3-TR cells infected with sh-AFAP1-AS1 or sh-NC were subcutaneously injected into nude mice followed by treatment with 3 mg/kg trastuzumab intraperitoneally once every two days for 20 days. The diameters of tumors were recorded twice a week using a caliper and tumor volume was calculated as (longest diameter) × (shortest diameter) 2 × 0.5. Then the mice were sacrificed to separate grafted tumors from them after 30 days and the weights of neoplasm were measured immediately after resection. Then, tissues were fixed for making pathological slides with 4% paraformaldehyde fixation followed by IHC staining for HER-2. Animal experiments were authorized by the Institutional Review Board of The First Affiliated Hospital of Zhengzhou University (Henan, China).

To experimentally construct lung metastases, SKBR-3-TR cells that had been transfected to stably express firefly luciferase (Xenogen Corporation, CA, USA) were infected with lentiviruses carrying control shRNA or sh-AFAP1-AS1. Single-cell suspension (2 × 10^6^ cells in 100 μl) in a total volume of 500 μL PBS containing 0.1% BSA was injected into the mouse lateral tail vein over a 60 s duration (five mice per group). After treatment with 1 mg/kg trastuzumab intraperitoneally once every two days for 5 weeks, mice were abdominally injected with luciferin (25 mg/ml in 0.1 ml PBS). At 15 min after injection, mice were anesthetized with phenobarbital sodium and lung metastases images were observed by IVIS-100 system (Xenogen). The bioluminescent images were overlaid on black and white photographs of the animals that were collected at the same time. Bioluminescence from relative optical intensity was defined manually.

### Bioinformatic analysis

The putative modification at the promoter of AFAP1-AS1 gene were predicted using (http://genome.ucsc.edu). Based on minimum free energy (MFE) and partition function, the stem-loop structure of AFAP1-AS1 was established by using (http://rna.tbi.univie.ac.at/).

### Western blot assay

The cells from all groups were collected, washed with 3 ml pre-cooling PBS, placed on ice and then boiled in SDS-sample buffer. Proteins samples were resolved by electrophoresing on 10% polyacrylamide gel electrophoresis (SDS-PAGE) and then transferred to polyvinylidene fluoride (PVDF) membrane. The membrane was blocked for 1 h with 5% skimmed milk at room temperature followed by incubation with the primary antibody against AUF1 (1:1000, Abcam, cat. no. ab61193), HER-2 (1:1000, Abcam, cat. no. ab16901), and GAPDH (1:5000, Abcam, ab9485) at 4 °C overnight and then incubated with corresponding secondary antibody at 37 °C for 1 h. The PVDF membrane was developed using ECL chemiluminescent reagent. Finally, the protein bands were performed with Bio-Rad Gel Doc XR+ system (Bio-Rad, Hercules, CA, USA).

### Statistical analysis

All experiments were performed in triplicate. Statistics were presented as mean ± SD. Comparison between two groups were analyzed using the Student’s t-test. One-way ANOVA was used for the comparison of multiple groups (> 2). Fisher exact testing was performed to evaluate the difference of proportions between different groups. A *P*-value < 0.05 was considered statistically significant for all analyses. Statistical analyses were performed using GraphPad Prism (v5.01, GraphPad Software Inc., San Diego, CA, USA). *P* < 0.05 was considered to indicate a statistically significant difference.

## Results

### LncRNA AFAP1-AS1 is upregulated in trastuzumab-resistant cells and activated by H3K27ac

In our previous study, breast cancer cells that are resistant to trastuzumab treatment, SKBR-3-TR and BT474-TR, were successfully established (Additional file 3: Figure S1a-b) [16]. By using SKBR-3-TR and SKBR-3 parental cells, we extended the sequencing samples based on the previous study [16]. Volcano plot was used for assessing gene expression variation between SKBR-3-TR and SKBR-3 cells (Fig. 1a). Genes with fold change more than 2 and false discovery rate less than 0.05 were identified as significantly differently expressed. The top 10 dysregulated lncRNAs are shown by hierarchical clustering analysis (Fig. 1b). We found that lncRNA AFAP1-AS1 was significantly dysregulated between the two types of cells. Interestingly, Yang et al. reported that AFAP1-AS1 was the most dysregulated lncRNA in HER-2-enriched subtype breast cancer [18]. Since HER-2 protein was the therapeutic target of trastuzumab, we hypothesized AFAP1-AS1 may be tightly linked with HER-2 expression and trastuzumab resistance. To confirm this assumption, we performed qRT-PCR to verify the expression of AFAP1-AS1 in breast cancer cells. As shown in Fig. 1c, AFAP1-AS1 was significantly upregulated in the established resistant sub-lines in contrast to the respective parental cell lines. Moreover, a significantly increased AFAP1-AS1 level was also verified in HER-2 positive breast cancer tissues in contrast to HER-2 negative tissues (Fig. 1d), which strongly supports our hypothesis.

**Fig. 1:** LncRNA AFAP1-AS1 is upregulated in trastuzumab-resistant cells and activated by H3K27ac. **a** Volcano plot images were drawn to show the differentially expressed genes between SKBR-3 and SKBR-3-TR cells. Five samples were used in each group. **b** The top 20 dysregulated lncRNAs were shown in heat map between SKBR-3 and SKBR-3-TR cells. **c** qRT-PCR was performed to measure the differential expression of AFAP1-AS1 in trastuzumab-resistant cells and parental sensitive cells, ^**^P < 0.01. **d** qRT-PCR showed that AFAP1-AS1 was upregulated in HER-2 positive patients compared to HER-2 negative patients. **e** The H3K27ac enriched area at the promoter of AFAP1-AS1 was predicted online at http://genome.ucsc.edu (shown as purple area). **f** RIP assay using anti-H3K27ac antibody showed that H3K27ac was enriched at the promoter region of AFAP1-AS1. Moreover, the enriched level was significantly increased in trastuzumab-resistant cells in contrast to parental sensitive cells, ^**^P < 0.01. **g** RIP assay showed that trastuzumab treatment increased the enrichment of H3K27ac at AFAP1-AS1 promoter in SKBR-3 and BT474 cells, ^*^P < 0.05, ^**^P < 0.01. **h** The acetyltransferase inhibitor, C646, significantly suppressed the binding level of H3K27ac, ^*^P < 0.05. **i** C646 treatment significantly inhibited the expression of AFAP1-AS1 in SKBR-3-TR and BT474-TR cells, ^*^P < 0.05

To identify the underlying mechanism by which AFAP1-AS1 was highly expressed in trastuzumab-resistant cells, we investigated the epigenetic modification sites at the promoter region of AFAP1-AS1. As shown in Fig. 1e, we identified a high enrichment of histone acetylation (H3K27ac) at promoter region of AFAP1-AS1 (*http://genome.ucsc.edu/*), suggesting that AFAP1-AS1 may be epigenetically activated by H3K27ac modification at promoter region. To prove this hypothesis, we performed ChIP assay. We verified that H3K27ac was enriched at the AFAP1-AS1 promoter region, and the enriched level was much higher in trastuzumab-resistant cells in contrast to respective parental cells (Fig. 1f). Moreover, trastuzumab treatment significantly increased the H3K27ac-enriched level in parental breast cancer cells (Fig. 1g). By using C646, a well-known acetyltransferase inhibitor, we found that C646 treatment repressed the H3K27ac enrichment and AFAP1-AS1 expression level (Fig. 1h and i). Taken together, we proved that AFAP1-AS1 was upregulated in trastuzumab-resistant cells, mainly due to the increased H3K27ac enrichment at AFAP1-AS1 promoter region.

### Silencing lncRNA AFAP1-AS1 reverses trastuzumab resistance

To determine the essential role of AFAP1-AS1 in trastuzumab resistance of breast cancer cells, we silenced AFAP1-AS1 in breast cancer cells. As shown in Fig. 2a, we observed a significantly decreased expression of AFAP1-AS1 in cells transfected with si-AFAP1-AS1#1 or si-AFAP1-AS1#2 compared to controlled cells. CCK8 assay revealed that knockdown of AFAP1-AS1 significantly increased the repression of cell viability induced by trastuzumab treatment (Fig. 2b and c). Moreover, the IC_50_ values of SKBR-3-TR and BT474-TR cells were dramatically decreased after knocking down of AFAP1-AS1 (Additional file 3: Figure S1c-d). It is known that trastuzumab exerts the anti-cancer effects via suppression of HER-2-regulated cancer proliferation and metastasis [19], herein we performed EdU staining and Transwell migration assay. EdU staining suggested that knockdown of AFAP1-AS1 significantly decreased cell proliferation (Fig. 2d and e). In addition, silence of AFAP1-AS1 decreased cell motility as evidenced by Transwell migration assay (Fig. 2f and g).

**Fig. 2:** Knockdown of AFAP1-AS1 reverses trastuzumab resistance of breast cancer cells. **a** AFAP1-AS1 was silenced by two specific small interfere oligonucleotides in SKBR-3-TR and BT474-TR cells, ^**^P < 0.01. **b-c** CCK8 assay revealed that knockdown of AFAP1-AS1 promoted trastuzumab-induced cell cytotoxicity. **d-e** EdU staining was performed to show the effect of AFAP1-AS1 knockdown in cell proliferation, ^*^P < 0.05. **f-g** Transwell migration assay was done to show the effect of AFAP1-AS1 on cell migration ability, ^**^P < 0.01. **h** qPCR verified the upregulation of AFAP1-AS1 after transduction of AFAP1-AS1-loaded plasmids in SKBR-3 and BT474 cells, ^***^P < 0.001. **i** CCK8 assay showed that overexpression of AFAP1-AS1 promoted cell viability, ^***^P < 0.001. **j-k** EdU staining showed that overexpression of AFAP1-AS1 increased cell proliferation in SKBR-3 and BT474 cells, ^*^P < 0.05. **l-m** Transwell assay showed that overexpression of AFAP1-AS1 promoted cell migratory ability, ^***^P < 0.001

We also investigated the influence of AFAP1-AS1 overexpression on trastuzumab resistance in SKBR-3 and BT474 parental cells. As shown Fig. 2h, AFAP1-AS1 was overexpressed in those cells after transduction of AFAP1-AS1-sequenced plasmids. By treating SKBR-3 and BT474 cells with trastuzumab (3 μg/ml for 48 h), we observed that enhanced AFAP1-AS abrogated the trastuzumab treatment-caused cell death when compared with control group (Fig. 2). Furthermore, AFAP2-AS1 increased proliferation and migration ability of SKBR-3 and BT474 cells (Fig. 2j-m).

### LncRNA AFAP1-AS1 level correlates with trastuzumab resistance in HER-2-positive breast cancer patients

qRT-PCR was performed to detect the expression of AFAP1-AS1 in tissue samples from 64 HER-2 positive patients (32 trastuzumab-resistant patients and 32 trastuzumab-responding patients according to iRECIST criteria). Figure 3a showed that AFAP1-AS1 was significantly upregulated in trastuzumab-resistant patients than in sensitive patients. To verify the predictive role of circulating AFAP1-AS1 in breast cancer patients, we examined whether AFAP1-AS1 was presented in extracellular milieu. As shown in Fig. 3b, expression of AFAP1-AS1 was detectable in serum of breast cancer patients and positively correlated with that in tissue samples. Serum AFAP1-AS1 level was significantly higher in non-responding patients compared to responding patients (Fig. 3c). When we divided the patients into high and low AFAP1-AS1 expressing groups (median value as cut-off), the proportion of responding patients was significantly lower in high AFAP1-AS1 level group than in low AFAP1-AS1 level group (Fig. 3d). We verified that distant metastasis was associated with high AFAP1-AS1 expression, while no significant difference was found in other clinical characteristics between AFAP1-AS1 high and low groups before trastuzumab therapy (Additional file 1, Table S1). Kaplan-Meier analysis showed that high AFAP1-AS1 levels in pretherapy serum were correlated with reduced PFS and OS in trastuzumab-treated breast cancer patients (Fig. 3e). Cox proportional hazards regression analysis further verified that high serumAFAP1-AS1 along with distant metastasis were an independent prognostic factor for breast cancer patients receiving trastuzumab treatment (Additional file 4, Table S3).

**Fig. 3:** High AFAP1-AS1 level was associated with poor response to breast cancer patients receiving trastuzumab treatment. **a** AFAP1-AS1 was upregulated in trastuzumab-resistant patients compared to patients responding to trastuzumab treatment, ^*^P < 0.05. **b** Pearson correlation testing identified a significant positive association between tissue AFAP1-AS1 and serum AFAP1-AS1 expression. **c** Serum AFAP1-AS1 level was increased in trastuzumab-resistant patients than in trastuzumab-responding patients, ^*^ P < 0.05. **d** The proportion of patients showing response to trastuzumab treatment was significant lower in high AFAP1-AS1 group than in low AFAP1-AS1 group. **e** Kaplan-Meier survival analysis showed that patients expressing high AFAP1-AS1 level had poorer overall survival and progressive-free survival

### Extracellular AFAP1-AS1 is transferred through incorporating into exosomes

To demonstrate whether extracellular AFAP1-AS1 confers trastuzumab resistance via incorporating into exosomes, we detected the existence pattern of intracellular and extracellular AFAP1-AS1. FISH assay with AFAP1-AS1 probe showed that AFAP1-AS1 was mainly distributed in cytoplasm of trastuzumab-resistant cells (Fig. 4a), suggesting that AFAP1-AS1 could be packaged into exosomes when secreted. Moreover, AFAP1-AS1 level in culture medium was unchanged upon treatment with RNase but significantly decreased when treated with RNase and Triton × 100 simultaneously, indicating that AFAP1-AS1 was wrapped with membrane instead of being released directly (Fig. 4b). To confirm this hypothesis, we isolated exosomes from culture medium. The representative micrograph and video taken by TEM showed vesicles with round or oval membrane (Fig. 4c, Additional file 5). NTA analysis revealed that the size of exosomes mostly ranges from 30 nm to 150 nm in diameter (Fig. 4d). Exosomes isolated from SKBR-3-TR cells and SKBR-3 parental cells exhibited similar morphology, size, and number. Western blot assay further verified that the exosome proteins, TSG-101 and CD81, were enriched in exosomes but not in cell extracts (Fig. 4e). In addition, the expression of exosomal AFAP1-AS1 levels were equal to that in extracellular AFAP1-AS1 levels in the cell culture medium, however, extracellular AFAP1-AS1 levels were almost eliminated after removing the exosomes from the medium (Fig. 4f), suggesting that exosome was the main carrier for extracellular AFAP1-AS1. Figure 4g showed that exosomal AFAP1-AS1 level was significantly higher in culture medium from trastuzumab resistant cell than that from sensitive cells.

**Fig. 4:** Extracellular AFAP1-AS1 is transferred through incorporating into exosomes. **a** RNA fluorescence in situ hybridization (RNA-FISH) verified that AFAP1-AS1 was mainly distributed in nuclear of SKBR-3-TR and BT474-TR cells. **b** Extracellular AFAP1-AS1 was degraded by treatment with RNAse A and Triton simultaneously, ^**^P < 0.01. **c** TEM scanning showed the exosomes images released by SKBR-3-TR and SKBR-3 cells. **d** Size distribution of exosomes were analyzed by Zetasizer. **e** Exosomal protein markers (TSG101 and CD81) detection by Western blot from purified exosomes and exosome-depleted cell extracts. **f** qRT-PCR analysis of lncRNA AFAP1-AS1 expression in exosomes, culture medium with or without exosomes, ^***^P < 0.001. **g** RT-qPCR analysis showed that exosomal AFAP1-AS1 was upregulated in trastuzumab-resistant cells in contrast to sensitive cells, ^**^P < 0.01. **h** RNA immunoprecipitation assay using anti-HNRNPA2B1 antibody showed that AFAP1-AS1 was associated with HNRNPA2B1 protein. **i** HNRNPA2B1 was silenced by specific oligonucleotides in both transcript and protein levels, ^**^P < 0.01. **j** Knockdown of HNRNPA2B1 decreased AFAP1-AS1 expression in SKBR-3-TR and BT474-TR cells, ^*^P < 0.05. **k** qRT-PCR and western blot verified the upregulation of HNRNPA2B1 by transfection of specific plasmids, ^**^P < 0.01. **l** AFAP1-AS1 was upregulated by overexpression of HNRNPA2B1 in SKBR-3-TR and BT474-TR cells, ^*^P < 0.05


**Additional file 5:** Dynamic video of exosome.


Then, we determined how AFAP1-AS1 is incorporated into exosomes. Previous study showed that RNA-binding protein, heterogeneous nuclear ribonucleoprotein A2B1 (HNRNPA2B1), is critical for packaging RNAs into exosomes [20]. To clarify whether HNRNPA2B1 is essential for AFAP1-AS1 loading into exosomes, we performed RIP assay with antibody against HNRNPA2B1. As shown in Fig. 4h, AFAP1-AS1 was pull down by HNRNPA2B1 antibody in SKBR-3-TR and BT474-TR cells. By silencing HNRNPA2B1, we found that exosomal AFAP1-AS1 was downregulated; whereas enhanced HNRNPA2B1 increased the expression of AFAP1-AS1 in exosomes accordingly (Fig. 4i-l). These data strongly suggest that AFAP1-AS1 was specifically packaged into exosomes in an HNRNPA2B1-dependent manner.

### Exosome mediated transfer of AFAP1-AS1 disseminates trastuzumab resistance

Take a step further, we proved the AFAP1-AS1contained in exosomes could be taken up by receipt cells via using two prolonged stages. First, we isolated exosomes from SKBR-3-TR cells and labelled with PKH26 dye followed by incubation with SKBR-3 and BT474 cells for 48 h. Figure 5a showed a strong red signal in receipt cells, indicating that the exosomes were taken up by recipient cells. Second, we examined whether these exosomes could deliver AFAP1-AS1 to recipient cells. By extracting cytoplasm RNA from receipt cells followed by qRT-PCR assay, we verified a significantly increased AFAP1-AS1 level in recipient parental cells upon incubation with exosomes from normal SKBR-3-TR cells, but not AFAP1-AS1-knockdown SKBR-3-TR cells (Fig. 5b). These results suggested that the AFAP1-AS1-contained exosomes can be taken by recipient cells.

**Fig. 5:** Exosome mediated transfer of lncRNAAFAP1-AS1 induces trastuzumab resistance. **a** Intercellular trafficking of exosomes among different cell lines by isolated exosomes labeled with PKH26 dye. **b** Treatment with exosomes derived from SKBR-3-TR increased AFAP1-AS1 level, however this effect was abrogated when SKBR-3-TR cells were silenced with AFAP1-AS1, ^*^P < 0.05. **c-d** CCK8 assay showed that SKBR-3-TR-derived exosomes induced trastuzumab resistance in SKBR-3 and BT474 cells, ^*^P < 0.05. **e** Nano-sight particle tracking analysis of the size distributions and number of exosomes from SKBR-3-TR cells treated with nSMase, GW4869. **f-g** CCK8 assay showed that incubation with exosomes from SKBR-3-TR cells treated with GW4869 failed to confer trastuzumab resistance to recipient cells. **h-i** CCK8 assay verified that knockdown of AFAP1-AS1(h) or HNRNPA2B1(i) inhibited the ability of co-cultured parental cells to acquire trastuzumab resistance

We further examined whether exosome-transferred AFAP1-AS1could confer the resistant phenotype to recipient cells. As shown in Fig. 5c-d, parental cells incubated with SKBR-3-TR-derived exosomes exhibited reduced sensitivity to trastuzumab treatment. To explore whether exosomes played a critical role in this effect, we reduced exosome production through the pharmacological inhibition of neutral sphingomyelinase-2 (nSMase) with GW4869 (Fig. 5e). As shown in Fig. 5f-g, incubation with culture medium from SKBR-3-TR cells treated with GW4869 failed to confer trastuzumab resistance to recipient cells. More importantly, knockdown of AFAP1-AS1 or HNRNPA2B1 suppressed the ability of co-cultured parental cells to acquire trastuzumab resistance (Fig. 5h and i).

### AFAP1-AS1 induces trastuzumab resistance via upregulation of HER-2 expression

Since we have proved the critical role of AFAP1-AS1 in trastuzumab resistance, we supposed that AFAP1-AS1 may be associated with HER-2 expression. By performing immunofluorescence assay, we detected in-situ HER-2 protein expression. HER-2 protein was upregulated in SKBR-3-TR and BT474-TR cells in contrast to the respective parental cells (Fig. 6a, Additional file 6: Figure S2a). Flow cytometry analysis showed that the percent of HER-2 positive cells in trastuzumab-resistant cells was significantly higher than that in parental cells (Additional file 6: Figure S2b-d). Then, we further examine whether HER-2 was regulated by AFAP1-AS1. As expected, knockdown of AFAP1-AS1 decreased HER-2 expression in trastuzumab-resistant cells (Fig. 6b). However, when we analyzed the expression of ERBB2 (*ERBB2 was used to indicate the coding RNA of HER-2 protein*) by performing qRT-PCR, the influence of AFAP1-AS1 on ERBB2 level was insignificant (Fig. 6c). In addition, increased AFAP1-AS1 upregulated HER-2 protein level (Fig. 6d) without influencing ERBB2 level (Fig. 2e). qRT-PCR also showed no correlation between AFAP1-AS1 and ERBB2 mRNA in breast cancer tissues (Additional file 6: Figure S2e). Together, we proved the role of AFAP1-AS1 in trastuzumab resistance and upregulation of HER-2 expression, however, whether AFAP1-AS1/HER-2 axis participated in trastuzumab resistance needs further confirmation.

**Fig. 6:** lncRNA AFAP1-AS1 regulates HER-2 protein level in breast cancer cells. **a** Immunofluorescence analysis of HER-2 protein in trastuzumab resistant cells and parental cells. **b** Western blot assay was performed to identify the effects of AFAP1-AS1 knockdown on HER-2 protein levels. **c** qRT-PCR showed that knockdown of AFAP1-AS1 had no influence on ERBB2 expression. **d** Overexpression of AFAP1-AS1 increased HER-2 protein level in SKBR-3 and BT474 cells. **e** Enhanced expression of AFAP1-AS1 showed no influence on ERBB2 expression

### LncRNA AFAP1-AS1 is associated with AUF1 to play critical roles

Our RNA-FISH showed that AFAP1-AS1 was mainly distributed in cytoplasm of trastuzumab-resistant cells (Fig. 4a). By conducting cellular fractionation PCR, we strengthened this conclusion (Fig. 7a). Similarly, subcellular distribution of AFAP1-AS1 was also mainly distributed in cytoplasm section of parental cell lines, SKBR-3 and BT474 (Additional file 7: Figure S3), suggesting that AFAP1-AS1 may regulate downstream pathways at post-transcriptional level. Moreover, no significant different distribution was observed between trastuzumab-resistant cells and parental sensitive cells, suggesting the formation of trastuzumab resistance was not due to the export or import nuclear of AFAP1-AS1. Based on online minimum free energy (MFE) evaluation (*http://rna.tbi.univie.ac.at/*), we predicted that AFAP1-AS1 transcript at the 911–1190 nt loci formed stem-loop structures (Fig. 7b), which is essential for the association with targeted RNA-binding proteins. To verify the proteins associated with AFAP1-AS1, RNA pulldown followed by mass spectrometry was performed, and several potential AFAP1-AS1-interacting proteins were identified (Additional file 8: Table S4), among which we identified AUF1, which could bind to 3′ untranslated region (UTR) of target mRNA and promote its translation without influencing the mRNA level [21]. Immunofluorescence assay showed co-expression in cytoplasm with AFAP1-AS1 (Fig. 7c). By designing AFAP1-AS1 probe and performing RNA pull-down assay, we found that AUF1 protein was enriched by AFAP1-AS1 (Fig. 7d). Moreover, RIP assay verified that AFAP1-AS1was precipitated by AUF1 antibody (Fig. 7e). AUF1 was not affected by AFAP1-AS1 knockdown in both transcript and protein levels (Fig. 7f). These suggest that AFAP1-AS1 is associated with AUF1 protein to play critical bio-functions.

**Fig. 7:** AFAP1-AS1 interacted with AUF1, thereby activated the translation of ERBB2. **a** Nuclear fraction experiment and qRT-PCR experiments were performed to detect the relative distribution of AFAP1-AS1 in nuclear and cytoplasm of SKBR-3-TR and BT474-TR cells. **b** Prediction of 911-1190 nt AFAP1-AS1 structure was based on minimum free energy (MFE) and partition function (http://rna.tbi.univie.ac.at/). **c** Immunofluorescence was performed to identify the subcellular distribution of AUF1 protein in SKBR-3-TR and BT474-TR cells. **d** RNA pulldown followed by western blotting was done with AFAP1-AS1 probe to verify the direct interaction between AUF1 and AFAP1-AS1. GAPDH served as internal control. **e** RIP was performed using anti-AUF1 and control IgG antibodies, followed by qRT-PCR to examine the enrichment of DANCR and U6. U6 served as negative control, ^***^P < 0.001. **f** qPCR showed that knockdown of AFAP1-AS1 showed no influence on AUF1 mRNA level. **g** Knockdown of AUF1 decreased HER-2 protein expression level without influencing the ERBB2 mRNA level. **h** Western blotting revealed that knockdown of AUF1 abrogated the increased HER-2 expression induced by overexpression of AFAP1-AS1. **i-j** The endogenous AUF1 binding to ERBB2 mRNA was increased by overexpression of AFAP1-AS1in SKBR-3 cells(i), while decreased by knockdown of AFAP1-AS1 in SKBR-3-TR and BT474-TR cells(j), ^*^P < 0.05, ^**^P < 0.01. **k** SKBR-3-TR and BT474-TR cells silenced with AFAP1-AS1 were cultured with 20 μg/ml Cycloheximide (CHX) for 0–60 min, then subjected to western blotting analysis

### LncRNA AFAP1-AS1 activates the translation of ERBB2 via recruiting AUF1

We sought to prove that AFAP1-AS1 increases translation activity of ERBB2 by binding with AUF1. Figure 7g showed that silence of AUF1 down-regulated HER-2 protein level without affecting ERBB2 level. Moreover, silence of AUF1 abrogated the AFAP1-AS1-inducedincrease of HER-2 protein in parental cells (Fig. 7h). To directly probe the essential role of AUF1, we performed RIP assay. Overexpression of AFAP1-AS1 increased endogenous AUF1 binding to ERBB2 in SKBR-3 cells while knockdown of AFAP1-AS1 exerted an opposite effect in trastuzumab-resistant cells (Fig. 7i and j). In addition, we treated trastuzumab resistant cells with cycloheximide (CHX), which inhibited the active synthesis and secretion of proteins. We measured the degradation of existing proteins and revealed that dysregulated AFAP1-AS1 had no effect on half-life of HER-2 protein (Fig. 7k), indicating that AFAP1-AS1 exerted no influence on HER-2 protein degradation. Hence, our results proved that AFAP1-AS1 guides AUF1 to binding to HER-2 mRNA, activating its translation without affecting the mRNA level.

### Knockdown of AFAP1-AS1 reverses trastuzumab resistance and metastasis in vivo

Based on our in vitro observations, we sought to validate our data by establishing xenografts in BALB/c nude mice models. We generated xenografts by subcutaneous injection of SKBR-3-TR and BT474-TR cells stably infected with sh-AFAP1-AS1 or sh-NC followed by intraperitoneal treatment of trastuzumab as described in Methods. By stripping tumors from nude mice, we presented the xenografts from different groups after 20 days of treatment (Fig. 8a). Moreover, the tumors formed in the sh-AFAP1-AS1 group were substantially smaller than those in the sh-NC group (Fig. 8b). By conducting IHC assay using anti-HER-2 antibody, we found that tumors formed from sh-AFAP1-AS1-infected cells exhibited decreased expression level of HER-2 than tumors formed from control cells (Fig. 8c).

**Fig. 8:** Knockdown of AFAP1-AS1 reversed trastuzumab resistance in vivo. **a** Representative images of the xenograft after intraperitoneal injection with once every 2 days 3 mg/kg trastuzumab treatment for 3 weeks in sh-NC or sh-AFAP1-AS1 cell groups. **b** Tumor sizes were calculated after injection every 2 days, ^***^P < 0.001 compared to sh-NC group. **c** Immunohistochemistry analysis revealed that the tumors developed from sh-AFAP1-AS1 cells displayed lower HER-2 staining than the sh-NC group. **d-e** Luciferase flux count (**d**) along with the visible number of metastases in lung (**e**) were significantly less in sh-AFAP1-AS1 group compared to sh-NC group. **f** Visualization of the HE-stained lung tissues from different sections

To confirm the role of AFAP1-AS1 in breast cancer metastasis, we injected SKBR-3-TR cells stably infected with sh-AFAP1-AS1 into tail veins of nude mice. By injecting single-cell suspension into the mouse lateral tail vein. As shown in Fig. 8d and e, the luciferase flux count along with the visible number of lung metastases formed by sh-AFAP1-AS1-infected cells were much less than the metastasis formed by sh-NC cells. HE-stained lung tissues showed significant improved positive areas in metastasis sections in contrast to normal lung sections (Fig. 8f). Altogether, we validated that silence of AFAP1-AS1 reversed trastuzumab resistance and metastasis of breast cancer in vivo.

## Discussion

It has now become widely accepted that mammalian genomes encode numerous lncRNAs [22]. Dysregulation of some lncRNAs has been shown in various type of cancers during cancer initiation, progression and chemoresistance, such as breast cancer [23]. However, the functions and mechanisms behind lncRNAs in breast cancer resistance, such as trastuzumab resistance, are still obscure. Based on our lncRNA microarray data, we identified an antisense lncRNA AFAP1-AS1, was highly expressed in trastuzumab-resistant cells than in parental cells. Gain and loss-functional assays revealed that knockdown of AFAP1-AS1 reverses trastuzumab resistance. In addition, extracellular AFAP1-AS1 confers trastuzumab resistance via incorporating into exosomes. Mechanistically, AFAP1-AS1 enhanced the translation of ERBB2 mRNA through binding with AUF1, thereby inducing the upregulation of HER-2 protein level and subsequent trastuzumab resistance (Fig. 9).

**Fig. 9:** A scheme of the proposed mechanisms. Trastuzumab treatment increases AFAP1-AS1 expression; which upregulates HER-2 expression by guiding AUF1 to activate the translation of ERBB2 mRNA, inducing trastuzumab resistance. In addition, extracellular AFAP1-AS1 from trastuzumab-resistant cells was packaged into exosomes and disseminates trastuzumab resistance in trastuzumab sensitive cells

Even more effective therapies using trastuzumab emtansine are now available [24]. Unfortunately, resistance to trastuzumab and other therapies that target the HER-2 pathway still occurs and some patients do not benefit from trastuzumab-based drug regimen. In addition, the identification of patients that will benefit from HER-2-directed therapies is greatly hindered by a lack of biomarkers for predicting therapeutic response [25]. This is despite the extensive retrospective analysis of phase III clinical trial data for the potential roles of related RTKs (i.e. EGFR, HER-3, IGF-1R), ligands (i.e. EGF, TGFα) or PI3K pathway alterations. The expression of HER-2 itself is currently the only biomarker to guide treatment decisions within this HER-2 positive patient cohort [26]. Therefore, numerous studies have been devoted to identifying the potential pathways and predictive biomarkers. At the same time, another newly developed anti-HER2 targeted antibody conjugate, Ado-trastuzumab emtasine (TDM-1), has emerged. It consists of trastuzumab plus the cytotoxic DM1 (emtasine), the first selectively and specifically delivering the second inside the HER2+ cancer cells through receptor-mediated endocytosis. It is specifically used for treatment of HER2+ breast cancer patients that have either received trastuzumab for metastatic disease or developed disease recurrence during trastuzumab treatment [27]. However, it is not experimentally proved whether T-DM1 could reverse trastuzumab resistance of breast cancer cells.

Functionally, dysregulation of lncRNAs is closely associated with aberrant biological behaviors of human cancers [28]. It is noteworthy some lncRNAs oriented in antisense direction with respect to a protein coding loci in the opposite strand usually act as regulators in many pathological processes [29]. Previous studies have shown that the natural antisense transcripts play critical roles in various physiological and pathological processes through regulating gene promoter activation and transcription [30–32]. One such recognized is lncRNA ZEB1-AS1, which epigenetically activates ZEB1 and promotes prostate cancer metastasis [33]. Previously, lncRNA AFAP1-AS1 was reported to act as a competing endogenous RNA of miR-423-5p to facilitate nasopharyngeal carcinoma metastasis [34]; while Yin et al. demonstrated that AFAP1-AS1 is associated with poor survival of patients with non-small cell lung cancer, and enhances cell proliferation via inhibition of p21 expression [35]. Until now, the exact regulatory mechanism of AFAP1-AS1 in cancer progression and resistance is not defined.

Our study investigated the potential function of AFAP1-AS1, and revealed that dysregulation of AFAP1-AS1 abrogated trastuzumab resistance. More importantly, we identified that extracellular AFAP1-AS1 could confer trastuzumab resistance through incorporating into exosomes. Exosomes are a new means of intercellular information exchange that have aroused great research interest [36]. Long neglected in research, exosomes were deemed nonfunctional cellular components to be discarded. However, it has been gradually revealed that exosomes are an important tool for the exchange of intercellular information and material [37]. Extracellular exosomes may spread drug resistance among heterogeneous populations of cancer cells, and ultimately inducing treatment failure of many cancer types [38]. However, the precise regulatory mechanism of how exosomes influence the tumor microenvironment for cell growth, metastasis and chemoresistance is largely unclear. By using a two-step validation, we verified that extracellular AFAP1-AS1 could confer trastuzumab resistance by incorporating into exosomes, which demonstrated a novel mechanism by which AFAP1-AS1 spread trastuzumab resistance.

Take a step further, we explored the downstream genes targeted by AFAP1-AS1. As trastuzumab suppressed breast cancer progression via the blockage of HER-2 signaling, we hypothesized AFAP1-AS1 may affect the expression of HER-2 protein. By conducting gain- or loss-functional assays, we proved that HER-2 was silenced by AFAP1-AS1 knockdown in trastuzumab resistant cells whereas upregulated by overexpression of AFAP1-AS1 in parental cells. More importantly, AFAP1-AS1 induced HER-2 protein level without influencing ERBB2 mRNA level. This indicates AFAP1-AS1 may regulate HER-2 protein at translational level. To uncover the underlying mechanism by which AFAP1-AS1 regulates HER-2 protein level, we screened the AFAP1-AS1-interacting proteins, and identified AUF1. AUF1 is a family of four RNA-binding proteins (RBPs) generated by alternative pre-messenger RNA (pre-mRNA) splicing, with canonical roles in controlling the stability or translation of mRNA targets based on recognition of AU-rich sequences within 3′ UTR of target mRNA [39]. Previously, Xiao et al. demonstrated that lncRNA FILNC1 represses c-Myc protein level by sequestering AUF1 from binding c-Myc mRNA and suppressing translation [40]. We validated that AUF1 was associated with AFAP1-AS1 and might act as an adaptor protein that cooperates with AUF1 to bind to ERBB2gene. By performing RIP assay, we revealed that AFU1 directly interacted with ERBB2, and AFAP1-AS1 increased this association level. Moreover, AFAP1-AS1 showed no effect on the HER-2 protein stability, which further supported our assumption.

Recent studies revealed the therapeutic potential of lncRNAs by designing specific silencing molecular or overexpression vector to knock off or upregulate the specific oncogenic lncRNAs in cancer, respectively [41]. Additionally, silencing nucleic acids against specific molecular targets may serve as new-generation therapeutic drugs to overcome the existed resistance [42]. Therefore, inhibition of trastuzumab resistance via precisely controlling AFAP1-AS1 levels might represent as potential therapeutic methods.

## Conclusion

We discovered that lncRNA AFAP1-AS1 confers trastuzumab resistance of breast cancer cells via packaging into exosomes. Mechanistically, AFAP1-AS1 promoted an AUF1-mediated activation of ERBB2 translation, causing an increased HER-2 expression and trastuzumab resistance. Uncovering the precise role of AFAP1-AS1/AUF1/HER-2 regulatory axis in trastuzumab resistance will not only increase our knowledge of noncoding RNAs-regulated therapeutic effect in cancer and the underlying regulatory mechanism, but also help develop more efficient strategies to reverse chemoresistance.

## Supplementary information

**Additional file 1: Table S1** Clinical characteristics of 64 HER2^+^ patients and the expression of AFAP1-AS1.

**Additional file 2: Table S2** Information of the qPCR primer sequences and silencing RNA sequences.

**Additional file 3: Figure S1** Determination of IC50 values of breast cancer cells. (a-b) The IC50 values of breast cancer parental cells (SKBR-3 and BT474) and established trastuzumab-resistant cells (SKBR-3-TR and BT474-TR) were determined via CCK8 assay. (c-d) The IC50 values of trastuzumab-resistant cells transfected with si-NC or si-AFAP1-AS1 were determined accordingly.

**Additional file 4: Table S3** Univariate and multivariate Cox proportional hazards regression model analysis of overall survival in breast cancer patients.

**Additional file 6: Figure S2** HER-2 protein was upregulated in trastuzumab-resistant cells. (a) Quantification of fluorescence intensity of Fig. 6a. (b-d) Flow cytometry analysis with anti-ERBB2 antibody (1:1000, ab31889, Abcam) showed a significantly elevated HER-2-positive cells in trastuzumab-resistant cells compared to sensitive cells, *P < 0.05. (e) Spearman correlation testing via qRT-PCR showed that no association was observed between AFAP1-AS1 and ERBB2 mRNA levels.

**Additional file 7: Figure S3** Nuclear fraction experiment and qRT-PCR experiments were performed to detect the relative distribution of AFAP1-AS1 in nuclear and cytoplasm of SKBR-3 and BT474 cells.

**Additional file 8: Table S4** Identification of AFAP1-AS1 binding proteins by MS.

## Data Availability

The datasets used and/or analyzed during the current study are available from the corresponding author on reasonable request.

## Abbreviations

ATCC: American Tissue Culture Collection
AUF1: AU-binding factor 1
ChIP: Chromatin immunoprecipitation
CHX: Cycloheximide
DAPI: 4’,6-diamidino-2-phenylindole
DMEM: Dulbecco’s modified Eagle medium
FBS: Fetal bovine serum
FISH: Fluorescence in situ hybridization
GAPDH: Glyceraldehyde 3-phosphate dehydrogenase
H3K27ac: H3K27 acetylation
HER-2: Human epidermal growth factor receptor 2
HNRNPA2B1: Heterogeneous nuclear ribonucleoprotein A2B1
IHC: Immunohistochemistry
lncRNAs: Long noncoding RNAs
MFE: Minimum free energy
NC: Negative control
OS: Overall survival
PBS: Phosphate-buffered saline
PCR: Polymerase chain reaction
PFS: Progressive-free survival
PVDF: Polyvinylidene fluoride
RIP: RNA immunoprecipitation
SD: Standard deviation
TEM: Transmission electron microscopy
UTR: Untranslated region
